# Effect of zinc nanoparticles seed priming and foliar application on the growth and physio-biochemical indices of spinach (*Spinacia oleracea* L.) under salt stress

This article has been retracted.

**DOI:** 10.1371/journal.pone.0263194

**Published:** 2022-02-22

**Authors:** Sara Zafar, Shagufta Perveen, Muhammad Kamran Khan, Muhammad Rashid Shaheen, Rashid Hussain, Nadeem Sarwar, Sahar Rashid, Muhammad Nafees, Ghulam Farid, Saud Alamri, Anis Ali Shah, Talha Javed, Mohammad Irfan, Manzer H. Siddiqui

**Affiliations:** 1 Government College University, Faisalabad, Pakistan; 2 Department of Horticultural Sciences, Faculty of Agriculture and Environment, The Islamia University of Bahawalpur, Bahawalpur, Punjab, Pakistan; 3 Nuclear Institute for Agriculture and Biology (NIAB), Faisalabad, Punjab, Pakistan; 4 Graduate School of Chinese Academy of Agricultural Sciences (GSCAAS), Beijing, China; 5 Horticultural Research Institute, Ayub Agricultural Research Institute, Faisalabad, Punjab, Pakistan; 6 Department of Botany and Microbiology, College of Science, King Saud University, Riyadh, Saudi Arabia; 7 Department of Botany, Division of Science and Technology University of Education, Lahore, Pakistan; 8 College of Agriculture, Fujian Agriculture and Forestry University, Fuzhou, China; 9 Plant Biology Section, School of Integrative Plant Science, Cornell University, Ithaca, NY, United States of America; Anhui Agricultural University, CHINA

## Abstract

Salt stress is the major risk to the seed germination and plant growth via affecting physiological and biochemical activities in plants. Zinc nanoparticles (ZnNPs) are emerged as a key agent in regulating the tolerance mechanism in plants under environmental stresses. However, the tolerance mechanisms which are regulated by ZnNPs in plants are still not fully understood. Therefore, the observation was planned to explore the role of ZnNPs **(**applied as priming and foliar) in reducing the harmful influence of sodium chloride (NaCl) stress on the development of spinach (*Spinacia oleracea* L.) plants. Varying concentrations of ZnNPs (0.1%, 0.2% & 0.3%) were employed to the spinach as seed priming and foliar, under control as well as salt stress environment. The alleviation of stress was observed in ZnNPs-applied spinach plants grown under salt stress, with a reduced rise in the concentration hydrogen peroxide, melondialdehyde and anthocyanin contents. A clear decline in soluble proteins, chlorophyll contents, ascorbic acid, sugars, and total phenolic contents was observed in stressed conditions. Exogenous ZnNPs suppressed the NaCl generated reduction in biochemical traits, and progress of spinach plants. However, ZnNPs spray at 0.3% followed by priming was the most prominent treatment in the accumulation of osmolytes and the production of antioxidant molecules in plants.

## Introduction

Salt stress obstructs the germination and development of plants. It causes a serious menace for agricultural production by affecting the plant nutrient uptake and disturbs their metabolic activities. About 45 million ha of the irrigated land is salt affected globally [1–3]. Salt stress affects plants by inhibiting their water uptake ability and deficiency of nutrients ultimately leading to the death of the plants [4]. Annual global loss in agriculture due to salt stress is 12 billion dollars and is increasing continuously [5, 6]. Salinity affects growth attributes, plant development, protein synthesis, metabolic activities like lipid metabolism, and carbohydrate metabolism [7]. Osmotic stress due to elevated amount of sodium (Na^+^) results in the shortage of water in plant cells thus affecting water potential [8]. Salinity is linked with toxicity in plants which is caused by excessive ions (Na^+^, Clˉ), oxidative & osmotic stress, nutritional disequilibrium, changes in metabolic activities, cell disorganization and distortion of membranes of the chloroplast, cell expansion and cell division reduction [9]. Salinity creates a harmful effect on the germination of seeds of many crops by forming an osmotic pressure on the outer side of the seed which inhibits water absorption [10]. It also adversely affects many processes of plants including photosynthesis, protein synthesis, lipid metabolism, and N-assimilation [11, 12]. To alleviate the harmful impacts of salinity, different methods are employed to maintain osmotic and ionic equilibrium to prevent plant damage [13, 14]. The methods commonly used are seed priming and foliar application; to alleviate the harmful effect of NaCl stress [15]. Priming boosts seed performance, uniformity, crop stand and improves yield under different environmental conditions and also helps to overcome dormancy. It induces changes in seed water content, cell cycle regulation, and seed ultrastructure modification [16]. Seed priming and foliar application alleviate stress responses during the development of seeds and establishment of seedlings [17]. Micronutrients priming and foliar application in the form of nanoparticles could be used in the development of crops to enhance their profit [18]. Zinc is an important nutrient. It maintains plant development, growth, health, and is beneficial for humans also. Zinc plays a dynamic role in protein metabolism, carbohydrate development, regulates IAA, acts as a major component of peptide enzymes, proteinases and dehydrogenases. It encourages seed maturation, production, and starch formation [19]. The use of specific amount of zinc nutrient coated by nanoparticles enhance grain yield with a rise in protein and a significant reduction in soluble sugar in wheat plants [20].

The nano-fertilization technique is a significant way to provide supplements slowly in a regulated way, which is vital to alleviate the challenges of fertilizers requirement [21]. This is due to the fact that micronutrients are transferred in the form of nanoparticles, that alter their chemical, and physical properties [22]. The deficiency of Zn causes disturbance in cell division, nitrogen metabolism, protein synthesis, photosynthesis, chlorophyll synthesis, reduction in the root, shoot, and dry matter, carbonic anhydrase function, integrity of membrane structure and function [23].

Zinc nanoparticles can be used as nano fertilizer. Nano fertilization enhances agriculture productivity and provide resistance against abiotic stresses. Nano fertilizers have encouraged a great interest to increase crop production. The profit margin of growers is increased by using nano fertilizers because it increases the yield and product quality [24].

Spinach (*Spinacia oleracea* L.) is a widely used leafy plant, its leaves and shoots serve the purpose of raw and boiled vegetables [25]. It can scavenge free radicals as it is rich in minerals, antioxidants, and vitamins like A, B, and C. It has several medical and food applications [26]. The plant has also several antibacterial compounds and folic acid which is useful for the treatment of anemia [27]. The current investigation focuses to find out the role and optimum concentration of Zinc nanoparticles (ZnNPs) on physio- biochemical characters of spinach plants under NaCl stressed environment.

## Materials and methods

The investigation (Table 1) was performed in the experimental area of Government College University Faisalabad, Pakistan, to examine the effect of priming and exogenic foliar treatment (0.1%, 0.2% and 0.3%) of zinc nanoparticles (ZnNPs) on spinach (*Spinacia oleracea* L.) (variety Desi) under normal and saline conditions. Foliar application of ZnNPs was done after 30 days. Plants were collected after two weeks of the exogenous foliar spray for physiological and biochemical analysis. Sodium chloride (100 mM NaCl) was used as a source of salt stress and ZnNPs by Sigma-Aldrich were used for priming and foliar treatment. The pots were filled with soil 7 kg each. About 10 seeds per pot were soaked in ZnNPs solution for 12 hours for priming purpose.

**Table 1:** Soil characteristics.

Texture	Loam	CO_3_^2-^ (meq/L)	Nil
ECe (dS/m)	2.04	HCO_3_ - (meq/L)	2.75
Ph	8.3	Zn (ppm)	2
Organic matter (%)	0.76	Available P (ppm)	3.1
Saturation	35	Available K^+^ (ppm)	80

### Determination of growth and physiochemical attributes

One plant randomly from every replicate was taken out gently, wholly clean with distilled water, and fresh weight of spinach shoot and root was noted in grams. The length of the shoot and root was recorded by using a measuring tape in cms. The same plant was put in a 65°C oven for 72 hours and the dry biomass was noted.

Chlorophyll analysis was done as proposed by Arnon [28]. Spinach leaves (0.5 g) were chopped into little pieces and immersed overnight in 80% acetone (10 ml) at about 4°C. The centrifugation of this mixture extract was done at 10,000 rpm for 5 minutes. After that a spectrophotometer (Hitachi-U2001, Tokyo, Japan) was used to measure absorbance of the supernatant at 480, 645 and 663 nm wavelengths.


$$\text{Chlorophyll}\;\text{a}\;({\text{mg}\;\text{g}}^{-1})=[12.7\left(\text{OD}\;663\right)-2.69\;\left(\text{OD}\;645\right)]\times \text{V}/1000\times \text{W}$$

$$\text{Chlorophyll}\;\text{b}(\text{mg}\;{\text{g}}^{-1})=[22.9\;\left(\text{OD}\;645\right)-4.68\;\left(\text{OD}\;663\right)]\times \text{V}/1000\times \text{W}$$

Total chlorophyll contents calculated by using this formula


$$\text{Total}\;\text{chlorophyll}\;(\text{mg}\;{\text{g}}^{-1})=\left[20.2\;\left(\text{OD}\;645\right)+8.02\;\left(\text{OD}\;663\right)\right]\times \text{V}/1000\times \text{W}$$

$$\text{Carotenoids}=\left\{\text{A}\;\text{Car}/\text{Em}\times 100\right\}\;\text{Where}\;\text{Em}\times 100=2500$$

$$\text{A}\;\text{Car}=\left[\left(\text{OD}\;480\right)+0.114\;\left(\text{OD}\;663\right)-0.638\;\left(\text{OD}\;645\right)\right]/2500$$

V = Volume of the extract (ml)

W = Weight of the fresh leaf (g)

OD = Optical density

Anthocyanin contents

About 0.5 g of leaves were homogenized in phosphate buffer (5 ml). The supernatant after centrifuge was taken in a quartz cuvette and the optical density (OD) was calculated at 600 nm wavelength [29].

### Antioxidant enzymes

Superoxide dismutase (SOD)

Giannopolitis & Ries [30] method was used to find out enzyme inhibition of the photochemical reduction of nitroblue tetrazolium (NBT). The absorbance was taken at 560 nm.

### Catalase (CAT) and peroxidase (POD)

About 0.5 g leaves were homogenised in phosphate buffer 50 mM of pH 7.8 in a cooled pestle and mortar using an ice bath, centrifuged at 12,000 x g for 15 minutes at 4 ˚C, and the supernatant was kept at -20 ˚C for CAT and POD enzyme activity analysis. Phosphate buffer (50 mM), H2O2 (5.9 mM), and 0.1 ml enzyme extract were used in the CAT reaction mixture. Every 20s, the optical density was measured at 240 nm. The reaction mixture for POD activity included 50 mM phosphate buffer, 20 mM guaiacol, 40 mM H2O2, and 0.1 ml enzyme extract. At 470 nm, the absorbance was measured every 20 seconds [31].

### Hydrogen peroxide (H_2_O_2_)

Fresh leaves weighing about 0.5 g were homogenized in 5 ml of 0.1 percent (w/w) trichloroacetic acid before being centrifuged for 15 minutes at 12,000 rpm. Phosphate buffer (pH 7.0) and potassium iodide were added to 0.5 ml of the reaction mixture. Vortex of this mixture was done and by using a UV visible spectrophotometer, measured its absorbance at 390 nm [32].

### Ascorbic acid contents (AsA)

Fresh leaves (0.5 g) were homogenized in a 10 ml solution of 6% trichloroacetic acid. The reaction mixture was centrifuged for 10 minutes at 10,000 rpm. The reaction mixture was heated for 20 minutes in a water bath containing 2 ml of the supernatant, 2 percent dinitrophenylhydrazine, and a drop of thiourea. Cooling brought the activity to a standstill. The optical density (OD) was measured at 520 nm after adding 5 ml of 80 percent sulphuric acid to the reaction mixture [33].

### Total soluble proteins

The Bradford method [34] was used to determine the total soluble proteins. In 10 ml of buffer, 0.5g of fresh leaves were crushed. The extract was centrifuged for 10 minutes at 10,000 rpm, with the temperature held at 4°C. The centrifugation was done and the suspension was stored at a cool place. In a test tube, combined 2 ml of Bradford reagent with 100 ul of the leaf extract and let for 15–20 minutes. At wavelength of 595 nm, absorbance was recorded.

### Total free amino acids

0.5 g of fresh leaves were crushed in 10 ml of phosphate buffer (0.05 M), at pH 7.8. The crushed sample was centrifuged at 10,000 rpm for 10 minutes at 4°C. In a test tube, the reaction mixture confined 0.5 ml of the extract, 0.5 ml of 4% ninhydrin and 0.5 ml of 2% pyridine. The test tubes containing a reaction mixture were vortexed. In a water bath, the test tubes were heated for 30 minutes at 100°C. Using a spectrophotometer, the optical density (OD) was recorded at 570 nm [35].

### Flavonoid contents

Leaves were homogenized in acetone. The reaction mixture comprised of 0.5 ml of extract, distilled water (2 ml), NaNO2 (5%, 0.6 ml), 10% aluminium trichloride (AlCl3, 0.5 ml) and 1M NaOH (2 ml). Gallic acid was taken as a standard. The absorbance was noted at 510 nm wavelength [36].

### Malondialdehyde (MDA) contents

The malondialdehyde (MDA) contents in spinach leaves were calculated by the protocol of Cakmak & Horst [37]. Fresh leaves 0.5 g were homogenized in 0.1% (w/w) trichloroacetic acid (TCA 10 ml) and were centrifuged for 12 min at 12,000 x g. 1 ml of supernatant wad added in 0.5% thiobarbituric acid that was made in 20% TCA. It was kept 25 min in a water bath at 95 ˚C, and the optical density was noted at 532 and 600 nm using a spectrophotometer.


$$\text{MDA}\;(\text{nmol}\;{\text{ml}}^{-1}\text{)}=\left[\left(\text{A}\;532–\text{A}\;600\right)/155,000\right]106.$$

### Statistical analysis

The data was evaluated by applying statistical software ‘Statistix 8.1’ to observe the significant differences between treatments. Complete randomized design (CRD) was used. The values of each treatment were compared by using the least significance difference test at a 5% level of significance.

## Results

Response of spinach to priming and foliar application of Zn nanoparticles under salt stress was observed in the study. Salinity significantly reduced morphological (Figs 1A–1F and 2A–2E) in spinach (Table 2). The priming and foliar application of Zn nanoparticles enhanced growth attributes such as biomass, root and shoot length, leaves per plant, and pigment analysis. Maximum fresh and dry weight was noted by the application 0.3% ZnNPs through seed priming and exogenous foliar spray under saline conditions followed by 0.2% ZnNPs. Shoot and root length significantly reduced under stress in spinach var. desi. However, priming of spinach seeds showed the highest shoot length at 0.2% ZnNPs under salt stress, while foliar application exhibited maximum value at 0.3% application under stress and non-stressed environment. Foliar treatment with ZnNPs exhibited maximum values of shoot and root length in comparison of priming application. Treatment of ZnNPs exhibited a positive effect on chlorophylls contents (Fig 2A and 2B). The highest Chla contents were observed by priming application of 0.3% ZnNPs under salt stress followed by 0.2% ZnNPs priming. A 27% decrease in Chlb contents was observed under NaCl stress in spinach var. Desi. Priming application of 0.2% ZnNPs increased 9.9% Chlb contents followed by 0.3% ZnNPs which exhibited 4.6% increase under salt stress. However, foliar application of 0.3% ZnNPs showed 5% increase under salt stress. Maximum Chlb content was observed at 0.3% ZnNPs by both priming (8.4%) and foliar (7.7%) application under salt stress. Priming application of 0.2% was more effectual in alleviating the detrimental effect of salt stress on carotenoid contents in spinach var. Desi (Fig 2D). The enhancement in the no. of leaves per plant was noted in spinach var. Desi by foliar application of 0.3% ZnNPs under salt stress (Fig 2E). Salinity stress and application of different concentrations of ZnNPs did not affect total soluble protein values significantly in spinach plants (Fig 3A). Total soluble sugars increased under salt stress however, the application of different levels of ZnNPs did not affect total soluble sugars significantly in spinach plants (Fig 3B). Treatment with ZnNPs improved total free amino acid content under salt stress. (Fig 3C). However, foliar use of ZnNPs enhanced TFA contents as compared to priming treatment under salt stress and decreased under non-stressed conditions. The study showed a decrease in phenolic contents under salt stress (Fig 3D). On the other hand, the treatment with ZnNPs enhanced the values of flavonoid and reducing sugars contents in spinach plants (Fig 3E and 3F). An enhancement in values of phenolic contents was observed with foliar use of ZnNPs as compared to priming treatment under salt stress. Regarding flavonoid contents values non-significantly differ under salt stress and with application of ZnNPs. Hydrogen peroxide and MDA contents significantly enhanced under salt stress in spinach plant (Fig 4). Application of ZnNPs non-significantly altered these oxidative stress attributes under saline conditions. Ascorbic acid contents decreased significantly under salt stress however, treatment of ZnNPs significantly enhanced ascorbic acid contents (Fig 4F). Foliar application of 0.3% ZnNPs was more effective in increasing ASA contents under salt stress. An enhancement in enzymatic antioxidant values was recorded under salt stress. However, 0.3% ZnNPs application maintained the activity under salt stress (Fig 4).

**Fig 1:** Effect of ZnNPs on growth attributes of spinach Desi variety under normal and saline conditions.

**Fig 2:** Effect of ZnNPs on pigment contents and number of leaves per plant of spinach variety Desi under normal and saline conditions.

**Fig 3:** Effect of ZnNPs on biochemical attributes of spinach variety Desi under normal and saline conditions.

**Fig 4:** Effect of ZnNPs on antioxidant activity of spinach variety Desi under normal and saline conditions.

**Table 2:** Mean square values for biochemical and yield attributes of spinach (*Spinaceae oleraceae* L.) plants with priming and foliar application of ZnNPs under saline conditions.

Source of variation	Salinity (S)	Treatment (T) ZnNPs	Salinity * Treatment	Error
Shoot Length	475.373***	24.506ns	5.246ns	13.3
Root Length	50.82*	8.088ns	2.983ns	7.381
Shoot fresh weight	1669.627***	114454ns	39.496ns	54.221
Root fresh weight	32.138***	4.494*	1.441ns	1.324
Shoot dry weight	17.012***	1.889*	1.189ns	0.701
Root dry weight	1.452***	0.232**	0.097ns	0.057
No. of leaves	64.381**	20.873*	5.381ns	6.929
Chl a	2.827***	0.069ns	0.057ns	0.035
Chl b	0039***	0.001ns	0.002ns	0.003
Chl t	3.529***	0.060ns	0.047ns	0.035
Carotenoids	3.975**	8.643ns	3.235ns	3.690
No. of leaves	64.381**	20.873*	5.381ns	6.929
Anthocyanin	42.681***	0.610ns	1.588ns	2.406
Total soluble proteins	6.512***	0.0583ns	0.042ns	0.083
Total soluble sugars	0.0079***	4.1522ns	6.675ns	4.796
Total free amino acids	0.345**	0.018ns	0.004ns	0.039
Phenolics	0.645ns	0.925ns	0.936ns	0.503
Flavonoid contents	0.014	0.013ns	0.022ns	0.009
Reducing sugars	47278.999ns	47099.906ns	47320.075ns	4.723
MDA	116.022***	1.077ns	0.479ns	9.643
CAT	10188.269***	82.879ns	813.617ns	517.357
POD	3446.346ns	38.686ns	182.530ns	961.884
SOD	2043.732ns	1392.351ns	2105.156ns	1004.179
H_2_O_2_	0.0013ns	0.0039*	0.0012ns	0.001
Ascorbic acid	14.081***	1.507*	0.865	0.506
*df*	1	6	6	28

*Df* degrees of freedom, ns nonsignificant, ***, **Significant at 0.001, 0.01 and *at 0.05 level of significance at 5% probability.

## Discussion

The research was performed to observe the outcomes of Zn nanoparticles seed priming and foliar application on the growth of spinach (*Spinacia oleracea* L.*)* under salt stress.

In the current investigation, salinity stress significantly lessened the growth and physiological traits of spinach plants as reported by Ibrahim et al. [38]. Spinach germination and development was critically reduced by salinity as shown by reduced fresh and dry weight of plants.

The decrease in growth under salt stress is due to osmotic stress. The uptake of nutrients and water is greatly affected under saline stress due to the reduced metabolic activity of plants. According to Xu et al. [39] fresh and dry biomass decreased under salt stress conditions. However, external use of ZnNPs enhanced the growth of spinach plants as shown in Fig 1. Similarly, ZnNPs induced growth improvement was reported in *Abelmoschus esculentus* [40]. The analysis of data exhibited that salinity stress reduced the chlorophyll content of spinach plants. However, carotenoids and anthocyanin contents increased under saline conditions in spinach plants. The findings are in accordance with Zafar et al. [41] in wheat. Total Chlorophyll was recorded highest at 0.1% foliar treatment of ZnNPs as stated by Sun et al. [42]. The decrease in photosynthetic pigment under salinity stress is also associated with the oxidation of chlorophyll contents through free radicals, interference of salt ions and pigment-protein complexes, chloroplasts disruption or enhancement in the values of chlorophyllase for the breakdown of chlorophyll [43, 44] as reported in *A*. *hybridus*. Shahbaz et al. [45] stated a stress-related decrease in Chl contents in wheat. In plants, the chlorophyll content amount is the main indicator for the study of their vigor to tolerate salinity [46, 47]. It has been recorded that zinc nano-fertilization enhance agriculture output and provide resistance against abiotic stresses such as NaCl stress [24]. The experiment shows highly positive results of ZnNPs on the spinach plants. Shoot and root length was recorded highest at 0.3% foliar application of ZnNPs as reported by Afrayeem et al. [48]. Similarly, shoot fresh and dry biomass were noted highest by 0.3% foliar application of ZnNPs as compared to priming treatments. Root fresh and dry weight was also recorded highest at 0.3% foliar application of ZnNPs as compared to priming treatments. The number of leaves was recorded maximum at 0.3% priming of ZnNPs as observed by Salama et al. [49]. It is stated by Ain et al. [50] and Itroutwar et al. [51] that application of ZnNPs is the best source of Zn fertilizer for growth.

The plants under saline conditions exhibited the maximum values of antioxidant enzymes as reported by Afrayeem et al. [48]. Under saline stress, ZnNPs helped to sustain SOD, POD, and CAT values. Plants antioxidant defense mechanism is activated by ZnNPs, which reduces oxidative stress damage [40]. H_2_O_2_ contents were also recorded highest under saline conditions as reported by Yusefi-Tanha et al. [52]. Malondialdehyde contents were recorded highest under saline conditions. However, exogenous treatment of ZnNPs lowered MDA levels, resulting in improved antioxidant response and membranes shielding role and enhances plant vigor to injury [41]. Flavonoids and total phenolic contents were recorded highest in plants at 0.3% priming treatment of ZnNPs under stress conditions. The same is reported by García-López et al. [53]. MDA contents were recorded maximum in salinity germinated plants as reported by Amooaghaie et al. [54]. Soluble sugars and total free amino acids were noted highest in plants under saline conditions. The results are reinforced by the work of Noreen et al. [55].

## Conclusion

Nano fertilizers have encouraged a great interest to increase the crop production. In the present experiment, salt stress impaired the growth and physio-biochemical attributes in spinach seedlings. However, treatment with ZnNPs suppressed the NaCl stress-induced reduction in biochemical attributes, and spinach plants growth. However, ZnNPs spray at 0.3% followed by priming was the most prominent treatment in the accumulation of osmolytes enzymatic and non-enzymatic antioxidant defense systems. Unlike conventional fertilizers, the fundamental economic benefits of nano fertilizers are efficient uptake and application in small quantities.
